RETRACTED

# G-Protein-Coupled Receptor Kinase-Interacting Protein 1 (GIT1) Promotes Head and Neck Squamous Cell Carcinoma Metastases via Activating the PI3K/AKT/mTOR Signal Pathway

**DOI:** 10.1155/2022/6881932

**Published:** 2022-01-25

**Authors:** Runze Xu, Ran Xu, Yuanxiang Wang, Weixing Wang, Lingling Jiang, Shishun Gong

**Affiliations:** ^1^Graduate School, Shanghai Jiaotong University School of Medicine, Shanghai 200025, China; ^2^Centre of Cancer Diagnosis and Treatment, JiangSu Rudong County People's Hospital, Nantong 226400, China; ^3^Department of Obstetrics and Gynecology, JiangSu Rudong Country People's Hospital, Nantong 226400, China; ^4^Department of Medical Nursing, JiangSu Rudong Country People's Hospital, Nantong 226400, China; ^5^Department of Rehabilitation, Hainan Medical College, Haikou, 571199 Hainan, China

## Abstract

**Objective:**

GIT1 is identified as a novel tumor oncogene in breast cancer. In this article, we aimed to explore the role of GIT1 in the progression of head and neck squamous cell carcinoma (HNSCC).

**Methods:**

GIT1 expression in HNSCC was detected by RT-qPCR, immunohistochemistry assay, and Western blot. HNSCC cell proliferation, migration, and invasion were examined by CCK-8 assay, Wound healing assay, and Transwell assay, respectively. Cell apoptosis was detected by flow cytometric analysis.

**Results:**

In our study, GIT1 was notably upregulated in HNSCC tissues and cells. Moreover, GIT1 expression level had positive corelation with pathological grade and nodal status of HNSCC. Functional experiments showed that knockdown of GIT1 restrained HNSCC proliferation, invasion, migration, and EMT and facilitated cell apoptosis. Furthermore, GIT1 knockdown was found to restrain HNSCC tumor growth and lung metastasis. Additionally, PI3K/AKT/mTOR signal pathway inhibitors suppressed the effect of GIT1 on HNSCC cell progression.

**Conclusion:**

GIT1 was upregulated in HNSCC and facilitated HNSCC cell progression by inducing PI3K/AKT/mTOR signal pathway. Therefore, we suggested that GIT1 might be a potential target for HNSCC treatment.

## 1. Introduction

Head and neck squamous cell carcinoma (HNSCC) is a type of malignant tumor originated from different organs of the head and neck [1, 2]. HNSCC is the sixth most common malignancy worldwide, and the eighth most common cause of cancer-related deaths [3]. The usual treatment for HNSCC patients is chemotherapy or radiotherapy [4, 5]. Despite extensive basic research and available options of clinical treatments, the 5-year survival rate of HNSCC patients is less than 50% [6]. Therefore, it is of great significance to explore the occurrence and development of HNSCC and develop new therapeutic targets to improve the prognosis of HNSCC patients.

RETRACTED

G-protein-coupled receptor kinase-interacting protein 1 (GIT1) is a cellular hetero shuttle protein that can interact with various protein kinases to regulate the overall cellular function [7]. The main function of GIT1 includes focal adhesion remodeling, receptor internalization, tyrosine kinase receptors, and signaling receptors [8]. Moreover, GIT1 expresses in the brain, liver, lung, thymus, and spleen and is involved in the regulation of various cellular processes [9]. Of note, GIT1 has been reported to promote bone regeneration by regulating ERK/NRF2 pathways in macrophages [10]. Dong et al. found that GIT1 was upregulated in breast cancer, and knockdown of GIT1 prevented cell growth, invasion, and migration [11]. In hepatocellular carcinoma, GIT1 promoted tumor progression by activating ERK/MMP9 pathway [12]. In addition, GIT1 was found to be upregulated in OSCC [13]. EMT is the initial step of tumor cell invasion and metastasis [14]. However, the effect of GIT1 on HNSCC tumor's multiplication and EMT progression *in vivo* is still unknown.

PI3K, the initiation of the PI3K/AKT/mTOR pathway, is activated by cell surface receptors to phosphorylation of downstream proteins, resulting a series of signal transduction [15]. The PI3K/AKT/mTOR pathway is negatively regulated through tumor inhibition of phosphatase on chromosome 10 in normal tissues, thus participating in dephosphorylation [16]. Singh et al. found that the PI3K/AKT/mTOR pathway inhibitors could improve gastric cancer deterioration [17]. Of note, PI3K/AKT/mTOR pathway was activated in hepatocellular carcinoma cells [18]. However, no systematic analysis of GIT1 on PI3K/AKT/mTOR pathway in HNSCC has been reported.

In this article, the effects of GIT1 on HNSCC cell growth and metastasis were probed. And we found that GIT1 facilitated HNSCC cell progression through PI3K/AKT/mTOR pathway. We suggested that GIT1 might be a tumor promoter in HNSCC and a potential target for HNSCC treatment.

## 2. Materials and Methods

### 2.1. Tissues Samples

88 HNSCC tissues were collected from JiangSu Rudong County People's Hospital. The experiment was approved by the Ethics Committee of JiangSu Rudong County People's Hospital (approval number: (2017) No. 033). All patients signed the informed consent.

### 2.2. Cell Culture

HNSCC cell lines FaDu, HN30, Cal27, SCC25, and HN8 and normal oral epithelial cell line HOK were from Shanghai Tongpai Biotechnology Co., Ltd. (Shanghai, China). HOK cells were cultured in HOK cell medium. FaDu, HN30, Cal27, and HN8 cells were cultured in DMEM medium with 10% FBS. SCC25 cells were cultured in DMEM/F12 medium at 37°C and 5% CO_2_.

RETRACTED

### 2.3. Plasmid Construction and Lentivirus Transfection

For GIT1 knockdown, shRNA was constructed by using pLenti6/BLOCKiT-DEST and named as sh-GIT1 or sh-NC, respectively. The target sequences in sh-GIT1 or sh-NC are as follows: sh-GIT1, 5′-GATCACAAGAATGGGCATT-3′; sh-NC, 5′-TTCTCCGAACGTGTCACGT-3′. HN8 and FaDu cells were transfected with sh-GIT1 or sh-NC lentivirus.

### 2.4. RT-qPCR

Total RNA was isolated via Trizol Reagent. Then, the cDNA was synthesized by SYBR Premix Ex Taq reagent kit. GIT1 expression was calculated by 2^−△△Ct^ method. GAPDH was the internal reference of GIT1. The primers are as follows: GIT1 forward: 5′-CCTCTTCCCAAAGAGGCCAG-3′, GIT1 reverse: 5′-TGAGTCAGCAGCTGGAAGTC-3′; GAPDH forward: 5′-CTCTGCTCCTCCTGTTCGAC-3′, GAPDH reverse: 5′-GACTCCGACCTTCACCTTCC-3′.

### 2.5. CCK-8 Assay

HNSCC cells were cultured in a 96-well plate at 37°C and 5% CO_2_. Then, after 24, 48, 72, and 96 h, CCK-8 reagent was added. Finally, the relative optical density (OD) was detected at 450 nm.

### 2.6. Wound-Healing Assay

HNSCC cells were added in a 6-well plate and grown in the complete medium until full confluence. Then, scratched the cells with a 10 *μ*L pipette tip and washed with DMEM medium to remove the detached cells. After 24 h, the wound areas were imaged by a microscopy.

### 2.7. Transwell Assay

Cells were added into the upper compartment with Matrigel. 500 *μ*L DMEM was added into the lower chamber. Then, 0.5% crystal violet was used to stained cells. Finally, the invaded cells were counted under an optical microscope.

### 2.8. Immunohistochemistry (IHC) Assay

First, paraffin sections were baked in an oven at 60°C for 30 min, then deparaffinized with xylene, ethanol, or PBS. Then, methanol with 0.3% H_2_O_2_ was used to quench the endogenous peroxidase activity for 5 min. PBS with 5% BSA was used to block the sides. After incubated with the primary antibodies, the secondary antibodies were incubated at 37°C for 30 min.

IHC scores were manually operated by two experienced pathologists according to the following formula: IHC score = staining intensity × amount of staining. The staining intensity scores are: 0, no staining; 1, weak staining; 2, moderate staining; 3, strong staining. The dyeing amount was classified as: less than 25% as 1; 25-75% as 2; greater than 75% as 3. Finally, multiply the two scores to get an overall score (on a scale of 1 to 9). The total score of 1-3 is defined as lower expression; 4-9 is defined as high expression.

### 2.9. Flow Cytometry Analysis

HNSCC cells (1 × 10^6^ cells/mL) were resuspended in the Binding Buffer (200 *μ*L), and detected by Annexin-V-FLUOS Staining Kit. The cells were gauged by a BD FACS Canto II Flow Cytometer.

RETRACTED

### 2.10. Western Blot Assay

Total protein samples were isolated with 10% SDS-PAGE, then transfected onto NC membrane. Next, the membrane was incubated with special primary antibodies overnight after blocked with 5% non-fat milk for 1 h. Then, membrane was incubated with secondary antibodies. The protein signals were measured by Western blotting substrate.

### 2.11. Animal Experiments

HN8-sh-NC or HN8-sh-GIT1 cells were injected into BALB/C nude mice subcutaneously. Then, mice were fed normally, and tumor volumes were gauged regularly. To explore the role of GIT1 in lung metastasis, FaDu-sh-GIT1 cells or FaDu-sh-NC cells were injected intravenously into BALB/C nude mice. The study was approved from the Animal Committee of JiangSu Rudong County People's Hospital ((2017) No. A-0541).

### 2.12. Statistical Analysis

The data were presented as mean ± SD. SPSS 20.0 and Graph Pad Prism 7.0. were used for data analysis. The differences between the two groups were evaluated by Student's *t*-test. The differences in multiple groups were evaluated by one-way ANOVA. When *p* < 0.05, it was considered statistically significant.

## 3. Results

### 3.1. GIT1 Was Markedly Overexpressed in HNSCC

First, to explore the expression of GIT1 in HNSCC, we searched the GEPIA dataset. The data displayed that GIT1 was expressed higher in HNSCC tissues than in normal tissues (Figure 1(a)). Furthermore, we assessed 88 HNSCC tissues by RT-qPCR assay. These data showed that GIT1 expression was notably overexpressed in HNSCC tissues (Figure 1(b)). As expected, the protein of GIT1 was highly expressed in HNSCC tissues (Figure 1(d)). Moreover, the protein of GIT1 was highly expressed in HNSCC cells (FaDu, HN30, SCC15, Cal27, SCC25, and HN8) compared with normal cells HOK (Figure 1(c)). Moreover, the GEPIA dataset displayed that there were no significant differences between GIT1 expression and the overall survival (OS) probability (*p* = 0.1, Figure 1(e)), while high GIT1 expression had a significant low disease-free survival (DFS) probability (*p* = 0.025, Figure 1(f)). The connection between GIT1 expression and clinicopathologic features was studied by IHC from 88 HNSCC specimens. As shown in Figure 1(g), the intensity of the staining was categorized as relatively weak (12/88), moderate (53/88), and strong (23/88) staining images (Figure 1(g)). Then, we divided 88 HNSCC patients into high GIT1 expression group and low GIT1 expression group. GIT1 expression has statistically significant correlation with pathological grades and nodal status of HNSCC (Table 1). Our data revealed that GIT1 might be participated in the progression of HNSCC.

RETRACTED

### 3.2. Knockdown of GIT1 Prevented Cell Proliferation and Induced Apoptosis in HNSCC

To detect the function of GIT1 in cell progression of HNSCC, we generated GIT1 knockdown cell lines from HN8 and FaDu cells with a lentivirus vector. The expression of GIT1 was effectively inhibited by sh-GIT1 (Figures 2(a) and 2(b)). Then, cell proliferation was assessed by the CCK-8 assay. GIT1 knockdown notably blocked the cell proliferation rate of HN8 and FaDu cells (Figures 2(c) and 2(d)). Furthermore, the cell apoptosis rate was found to be notably increased by GIT1 knockdown in HN8 and FaDu cells (Figure 2(e)). Our findings demonstrated that GIT1 knockdown restrained proliferation and facilitated cell apoptosis in HNSCC.

### 3.3. Knockdown of GIT1 Restrained Cell Migration, Cell Invasion, and EMT in HNSCC Cells

Furthermore, the effect of GIT1 on cell invasion and migration was investigated by Transwell assay and wound healing assay. GIT1 knockdown remarkably repressed the migration viability of HN8 and FaDu cells (Figure 3(a)). GIT1 knockdown reduced the number of invasive cells in HN8 and FaDu cells (Figure 3(b)). Moreover, GIT1 knockdown decreased the protein expression of N-cadherin and Vimentin, while facilitated the protein expression of E-cadherin in HN8 and FaDu cells (Figure 3(c)). Therefore, the data indicated that GIT1 knockout repressed cell metastasis and blocked EMT progression of HNSCC cells.

### 3.4. Knockdown of GIT1 Inhibited HNSCC Tumor Growth and Metastasis *In Vivo*

To detect the role of GIT1 on tumor growth, HN8 cells with GIT1 knockdown was injected into the tail vein of nude mice. The tumor weight and volume in sh-GIT1 group were markedly suppressed compared with sh-NC group (Figures 4(a) and 4(b)). Moreover, after inoculation for 30 days, tumors were lighter in sh-GIT1 group than in sh-NC group (Figure 4(c)). The results indicated that GIT1 knockdown inhibited tumor growth *in vivo*.

To confirm the important role of GIT1 in lung metastasis, Fadu cells transfected with GIT1 silencing were injected into nude mice. After 4 weeks, the lungs were dissected out for IHC staining analysis. The lung metastatic nodules in mice GIT1 knockdown group was markedly reduced (magnification 40х, Figures 4(d) and 4(e)). These data revealed that GIT1 knockdown prevented HNSCC lung metastasis in vivo.

### 3.5. GIT1 Regulated Cell Progression by Regulating PI3K/AKT/mTOR Pathway

To explore the specific mechanism of GIT1 in HNSCC cell progression, GIT1 overexpression or GIT1 knockdown was transfected into SCC25 cells. GIT1 knockdown reduced the protein expression of p-PI3K, p-Akt, and p-mTOR (Figure 5(a)). Inversely, GIT1 overexpression increased the protein expression level of p-PI3K, p-Akt, and p-mTOR (Figure 5(a)). Furthermore, HN8 cell and FaDu-transfected cell overexpression GIT1 were treated with P13K inhibitor (LY290004). The cell proliferation was notably promoted by GIT1 overexpression, while inhibited by LY290004 (Figures 5(b) and 5(c)). Similarly, LY290004 inhibited the effect of GIT1 on cell metastasis in HN8 and FaDu cells (Figures 5(d) and 5(e)). Besides that, LY290004 inhibited the effect of GIT1 on EMT progression in HN8 and FaDu cells (Figure 5(f)). Collectively, our data suggested that GIT1 promoted HNSCC cell progression by activating PI3K/AKT/mTOR pathway.

RETRACTED

## 4. Discussion

In the current study, we highlighted the expression and regulatory effect of GIT1 in HNSCC. We noticed that GIT1 was notably upregulated in HNSCC patients. Functionally, our results demonstrated that GIT1 knockdown restrained cell metastasis and EMT and promoted cell apoptosis in HNSCC cells. Previous studies have showed that GIT1 drived tumor progression in osteosarcoma [19]. Zhao et al. discovered that MeCP2 facilitated cell growth by upregulating GIT1 expression in gastric cancer [20]. In osteosarcoma, GIT1 was discovered to be highly expressed, and GIT1 knockout repressed cell invasion, cell growth, and angiogenesis [21]. Consistent with our findings, GIT1 knockout was confirmed to inhibit tumor growth in breast cancer [11, 22]. In oral squamous cell carcinoma, GIT1 silencing inhibited cell migration, invasion, and lung metastasis [13]. Similarly, GIT1 knockdown also suppressed tumor growth and lung metastasis in vivo. Of note, GIT1 has strong correlation with the pathological grade and nodal status in HNSCC. Chang et al. found that GIT1 was related to the poor prognosis of patients with non-small-cell lung cancer [23]. Consequently, our study indicated that GIT1 plays an oncogenic role in the progression of HNSCC.

In recent years, PI3K/AKT/mTOR pathway has been found to play a crucial role in tumor progression. For example, CD47 was found to function as an oncogene by activating PI3K/AKT/mTOR pathway in endometrial carcinoma [24]. Moreover, previous research findings have indicated that the PI3K/AKT/mTOR pathway is activated in 90%-100% of HNSCC [25]. In the current work, we found that the inhibition of the PI3K/AKT/mTOR prevented the function of GIT1 on proliferation, metastasis, and EMT progression in HNSCC. Choi et al. found that adenosine induced cell apoptosis by blocking the phosphorylation levels of PI3K/AKT/mTOR in FaDu cells [26]. Similarly, the PI3K/AKT/mTOR pathway was over activated in head and neck cancer [27] and hepatocellular carcinoma [18]. Hence, we suggest that GIT1 promoted HNSCC cell progression through activating PI3K/AKT/mTOR pathway.

RETRACTED

## 5. Conclusion

In sum, we have shown that GIT1 is closely associated with poor prognosis in HNSCC patients and facilitates cell growth, metastasis, and EMT by upregulating PI3K/AKT/mTOR signaling pathway. Hence, our findings suggest that GIT1 may be a therapeutic target for HNSCC.

## Figures and Tables

**Figure 1:** GIT1 was markedly upregulated in HNSCC tissues and cell lines and associated with poor prognosis in HNSCC. (a) GEPIA dataset showed that GIT1 was upregulated in 519 HNSCC tissues relative to 44 normal tissues. (b) GIT1 was higher expressed in HNSCC tissues than in normal tissues. (c) The protein expression of GIT1 was increased in HNSCC cell lines (HN30, HN8, Cal-27, SCC25, and FaDu) compared with in HOK cells. (d) The protein expression of GIT1 was obviously higher in HNSCC tissues than in normal tissues. (e) GEPIA dataset displayed that GIT1 expression had no significance on OS probability of HNSCC patients. (f) GEPIA dataset displayed that high GIT1 expression had a significant low DFS probability. (g) IHC assay of GIT1 expression in tissues microarrays was shown (relatively weak, moderate, and strong staining). ^∗∗^*p* < 0.01.

**Figure 2:** Knockdown of GIT1 prevented cell proliferation and induced cell apoptosis in HNSCC. (a) The protein expression of GIT1was significantly declined in HN8 cells transfected with GIT1 knockdown. (b) The protein expression of GIT1was significantly declined in FaDu cells transfected with GIT1 knockdown. (c, d) GIT1 knockdown obviously inhibited cell proliferation in HN8 and FaDu cells. (e) GIT1 knockdown significantly promoted cell apoptosis in HN8 and FaDu cells. ^∗^*p* < 0.05, ^∗∗^*p* < 0.01.

**Figure 3:** Knockdown of GIT1 restrained cell migration, cell invasion, and EMT of HNSCC cells. (a) GIT1 knockdown inhibited cell migration ability in HN8 and FaDu cells. (b) GIT1 knockdown suppressed cell invasion ability in HN8 and FaDu cells. (c) GIT1 knockdown suppressed the EMT progression in HN8 and FaDu cells. ^∗∗^*p* < 0.01.

**Figure 4:** Knockdown of GIT1 inhibited HNSCC tumor growth and metastasis in vivo. (a) Mice were killed and the tumors were isolated. (b) The tumor volumes were measured on the indicated days. (c) One month after cell injection, the average tumor weight was measured. (d) H&E staining showed the lung metastatic nodules. (e) The number of lung metastatic nodules in the mice GIT1 knockdown group was markedly reduced compared to the GIT1 control group. ^∗^*p* < 0.05, ^∗∗^*p* < 0.01.

**Figure 5:** GIT1 affected cell progression by regulating PIK3/AKT/mTOR pathway. (a) GIT1 knockdown diminished the protein expression level of p-P13K, p-Akt, and p-mTOR. GIT1 overexpression increased the protein expression level of p-PI3K, p-Akt, and p-mTOR compared with in control group. (b, c) GIT1 overexpression significantly promoted cell proliferation, while LY290004 weakened the effect of GIT1 on cell proliferation in HN8 and FaDu cells. (d) GIT1 overexpression obviously promoted cell migration ability, while LY290004 weakened the effect of GIT1 on cell migration ability in HN8 and FaDu cells. (e) GIT1 overexpression obviously promoted cell invasion ability, while LY290004 weakened the effect of GIT1 on cell invasion ability in HN8 and FaDu cells. (f) GIT1 overexpression obviously promoted EMT progression, while LY290004 weakened the effect of GIT1 on EMT progression in HN8 and FaDu cells. ^∗∗^*p* < 0.01, compared with vector group; ^##^*p* < 0.01, compared with GIT1 group.

RETRACTED

**Table 1:** Correlations between GIT1 levels and clinical characteristics in HNSCC patients.

Clinical characteristics	Number of cases	GIT1 expression		*p* value
	*n* = 88	Low (*n* = 39)	High (*n* = 49)	
Age (years)				0.275
>65	35	18	17	
≤65	53	21	32	
Gender				0.094
Male	58	22	36	
Female	30	17	13	
Tumor size				0.906
T1/2	40	18	22	
T3/4	48	21	27	
Smoking				0.516
Yes	28	11	17	
No	60	28	32	
Drinking				0.740
Yes	31	13	18	
No	57	26	31	
Pathological grade				0.027^∗^
I-II	29	31	28	
II-III	29	8	21	
Nodal status				0.008^∗∗^
N0	38	23	15	
≥N1	50	16	34	

^∗^ *p* < 0.05, ^∗∗^*p* < 0.01 the difference is significant. LDH: lactate dehydrogenase; IPI: international prognostic index.

## Data Availability

The data used to support the findings of this study are available from the corresponding author upon request.
